The article "Designing of an mRNA vaccine against high-risk human papillomavirus targeting the E6 and E7 oncoproteins exploiting immunoinformatics and dynamic simulation" was retracted in 2025. Reasons: compromised peer review; unreliable results or conclusions.

# Designing of an mRNA vaccine against high-risk human papillomavirus targeting the E6 and E7 oncoproteins exploiting immunoinformatics and dynamic simulation

**DOI:** 10.1371/journal.pone.0313559

**Published:** 2025-01-06

**Authors:** Md. Mijanur Rahman, Md. Habib Ullah Masum, Rehana Parvin, Shuvo Chandra Das, Asma Talukder

**Affiliations:** 1 Department of Microbiology, Noakhali Science and Technology University, Noakhali, Bangladesh; 2 Microbiology, Cancer and Bioinformatics Research Group, Noakhali Science and Technology University, Noakhali, Bangladesh; 3 School of Pharmacy and Medical Sciences, Griffith University, Queensland, Australia; 4 Department of Genomics and Bioinformatics, Faculty of Biotechnology and Genetic Engineering, Chattogram Veterinary and Animal Sciences University, Khulshi, Chittagong, Bangladesh; 5 Department of Pathology and Parasitology, Faculty of Veterinary Medicine, Chattogram Veterinary and Animal Sciences University, Khulshi, Chittagong, Bangladesh; 6 Department of Biotechnology and Genetic Engineering, Noakhali Science and Technology University, Noakhali, Bangladesh; University of Chittagong, BANGLADESH

## Abstract

Human papillomavirus 16 and human papillomavirus 18 have been associated with different life-threatening cancers, including cervical, lung, penal, vulval, vaginal, anal, and oropharyngeal cancers, while cervical cancer is the most prominent one. Several research studies have suggested that the oncoproteins E6 and E7 are the leading cause of cancers associated with the human papillomavirus infection. Therefore, we developed two mRNA vaccines (V1 and V2) targeting these oncoproteins. We used several bioinformatics tools to predict helper T lymphocyte, cytotoxic T lymphocyte, and B-cell epitopes derived from the proteins and assessed their antigenicity, allergenicity, and toxicity. Both vaccines were constructed using selected epitopes, linkers, and adjuvants. After that, the vaccines were applied for physicochemical properties, secondary and tertiary structure predictions, and subsequent docking and simulation analyses. Accordingly, vaccine 1 (V1) and vaccine 2 (V2) showed better hydrophilicity with the grand average hydropathicity score of -0.811 and -0.648, respectively. The secondary and tertiary structures of the vaccines were also deemed satisfactory, with high stability indicated by the Ramachandran plot (V1:94.5% and V2:87.1%) and Z scores (V1: -5.15 and V2: -4.1). Docking analysis revealed substantial affinity of the vaccines towards the toll-like receptor-2 (V1: -1159.3, V2: -1246.3) and toll-like receptor-4 (V1: -1109.3, V2: -1244.8) receptors. Molecular dynamic simulation validated structural integrity and indicated varying stability throughout the simulation. Codon optimization showed significant expression of the vaccines (V1:51.88% and V2:51.63%) in *E*. *coli* vectors. Furthermore, regarding immune stimulation, the vaccines elicited significant B-cell and T-cell responses, including sustained adaptive and innate immune responses. Finally, thermodynamic predictions indicated stable mRNA structures of the vaccines (V1: -502.60 kcal/mol and V2: -450.90 kcal/mol). The proposed vaccines designed effectively targeting human papillomavirus oncoproteins have demonstrated promising results via robust immune responses, suggesting their suitability for further clinical advancement, including *in vitro* and *in vivo* experiments.

The article "Designing of an mRNA vaccine against high-risk human papillomavirus targeting the E6 and E7 oncoproteins exploiting immunoinformatics and dynamic simulation" was retracted in 2025. Reasons: compromised peer review; unreliable results or conclusions.

## Introduction

Human papillomaviruses (HPVs) are small double-stranded DNA viruses belonging to the papillomaviridae family that cause infections in human mucous epithelia. It is the most frequent sexually transmitted disease (STD) worldwide [1]. HPV has been associated with 5% of cancer cases, affecting various parts of the human body, including the lung, cervix, penis, vulva, vagina, anus, and oropharynx, and thereby associated with cervical, penal, vulval, vaginal, anal, and oropharyngeal cancer [2–5]. Additionally, there is evidence suggesting the involvement of HPV in conjunctival malignancies [3]. Cervical cancer is the most significant form of cancer caused by human HPV; more than 95% of cervical cancers have been associated with HPV [2]. According to the World Health Organization (WHO), it holds the 14th position among all types of cancers and is the 4th most prevalent cancer among women globally [6, 7]. Annually, an estimated 500,000 cases of cervical cancer have been identified, where nearly half of which are fatal [8]. The prevalence of STDs among young women typically ranges from around 30%, but in some demographics, it may reach as high as 64%. Interestingly, 50% of young women had contracted a cervical HPV infection within four years of their first sexual contact [9]. There is an enormous variation in the burden of cervical disease, with more than 85% of cases and fatalities occurring in countries with low and moderate incomes [10]. These disparities are mostly attributable to inadequate cervical cancer screening and treatment strategies [11]. Over the last several decades, a combination of surgery, radiation therapy, chemotherapy, and, more recently, immunotherapy have become the mainstay of cervical cancer treatment. Currently, the United States Food and Drug Administration (US-FDA) has approved three immunotherapy alternatives for treating cervical cancer, including Bevacizumab, Tisotumab vedotin, and Pembrolizumab [12]. However, these strategies lack efficacy, are highly costly, and, more importantly, have adverse effects, including fever, headache, skin rashes or itching, abdominal pain, nausea, cough, diarrhea, constipation, fatigue, loss of appetite, peripheral neuropathy, and hypothyroidism [13–15]. Hence, vaccination is the only practical approach for minimizing the risks of developing cervical cancer as well as for its prevention.

The article "Designing of an mRNA vaccine against high-risk human papillomavirus targeting the E6 and E7 oncoproteins exploiting immunoinformatics and dynamic simulation" was retracted in 2025. Reasons: compromised peer review; unreliable results or conclusions.

Meanwhile, up to 70% of oropharyngeal cancers have been attributed to HPV, and the incidence of oral squamous cell carcinomas (OSCCs) in both Europe and North America is on an upward trajectory [16]. Oropharyngeal cancers now surpass cervical cancer events in the United States and are the leading cancer associated with HPV [17]. Although there is still uncertainty about the involvement of HPV in oropharyngeal cancers, it is possible to identify HPV in a specific subset of these malignancies [18, 19]. There was a statistically significant association between increasing levels of anti-HPV-16 IgG antibody and oropharyngeal cancer, based on research conducted in South Africa [20]. The yearly worldwide frequency of squamous cell carcinoma of the anus caused by HPV was estimated to be 30,416 cases, while women accounted for two-thirds of these cases [21].

Currently, more than 200 strains of HPV have been identified, which belong to 29 genera, with most of them infecting humans [22]. Around half of these strains target the epithelium of the female genitalia. However, there are two types of genital papillomaviruses: low-risk and high-risk. Low-risk HPVs cause benign lesions, while high-risk HPVs can develop malignant lesions [23, 24]. Notably, many cervical cancers are found to have DNA from high-risk types of HPV [25, 26], and HPV 16 and HPV 18 have been reported as the leading cause of cervical cancer. The two transforming proteins (E6 and E7) encoded by these strains, function through their associations with the tumor suppressor proteins p53 and retinoblastoma (Rb), respectively [27]. The continual expression of E6 and E7 in tumors and derived cell lines, even years after the initial immortalizing events, reveals their crucial role in sustaining the altered phenotype [27, 28]. The immortalization of primary human keratinocytes requires the symbiotic actions of E6 and E7, with E6 blocking cell survival pathways and E7 encouraging cell proliferation [28, 29]. As part of the ubiquitin proteolytic process, E6 interacts with an accessory protein called E6-AP, allowing it to degrade p53 [30, 31]. On the other hand, the E7 proteins from high-risk HPVs have an affinity for Rb [32, 33] and other pocket proteins like p107 and p130 [34, 35], resulting in altered functions of these cell cycle regulators. While low-risk E7 proteins bind Rb with significantly lower affinities, low-risk E6 proteins cannot abolish p53 functions [36]. It has also been suggested that p53 plays a crucial role in preserving the stability of the genome. However, the E6 of the high-risk types inhibits all of these functions of p53, thus leading to uncontrolled cell cycle and cell immortalization [37, 38]. The role of the Rb gene, along with p53, is crucial in regulating the cell cycle and its checkpoints. During the S phase, the protein Rb forms a complex with the transcription factor E2F, thus phosphorylating itself and causing E2F to be released, which is necessary for DNA synthesis [39]. However, the interaction between E7 and Rb prevents the binding of Rb to E2F, leading to persistent activation of E2F and subsequent expression of the associated genes [40].

The article "Designing of an mRNA vaccine against high-risk human papillomavirus targeting the E6 and E7 oncoproteins exploiting immunoinformatics and dynamic simulation" was retracted in 2025. Reasons: compromised peer review; unreliable results or conclusions.

There are currently six authorized alternatives in the landscape of HPV vaccines, all of which fall under the category of virus-like particle (VLP) vaccines, including Cervarix^®^, Cecolin^®^, WalrinvaxV, GARDASIL^®^, Cervavac^®^, and GARDASIL9^®^ [41]. Nevertheless, although VLPs imitate viral structures, they do not possess genetic material for replication. This could result in less effective immune responses, especially in susceptible groups such as the elderly or those with weakened immune systems [41]. Considering these factors, mRNA-based therapeutics may address these challenges while improving the management of infectious diseases and cancer [42, 43]. Non-infectious and non-integrating mRNA vaccines offer advantages over conventional immunizations. Several mRNA vaccines have been designed targeting HPV, which also showed promising outcomes in clinical and pre-clinical trials [44–47].

With the advent of immunoinformatics tools, computational approaches for vaccine design have become more widespread in the post-genomics era [48, 49]. Immunoinformatics is a revolutionary strategy that offers many advantages for vaccine development [49–51]. It utilizes machine learning algorithms to promptly analyze substantial amount of structural, genomic, and proteomic data to identify prospective vaccine candidates [52, 53]. This approach facilitates the prediction of immune-stimulating epitopes and antigenic targets, optimizing vaccine component selection for enhanced safety and efficacy [49, 54]. This precision-oriented approach reduces the need for rigorous and expensive clinical trials, exploiting resources and expediting vaccine production schedules [52, 55]. Yet, a few hurdles need to be explored before applying immunoinformatics in vaccine manufacturing. Immunoinformatics depends on extensive data, yet data quality and quantity discrepancies may affect the precision of vaccine target predictions. Moreover, predicted targets may not reliably elicit intended immune responses or may provoke adverse effects [55–57]. Leveraging immunoinformatics in vaccine development requires interdisciplinary alliance, technological advancements, and continual research to address the challenges [53]. This research used immunoinformatics approaches to identify prospective vaccine targets from the proteome of HPV.

The article "Designing of an mRNA vaccine against high-risk human papillomavirus targeting the E6 and E7 oncoproteins exploiting immunoinformatics and dynamic simulation" was retracted in 2025. Reasons: compromised peer review; unreliable results or conclusions.

This work focuses on the immunoinformatics for developing mRNA vaccines to address the urgent public need for HPV vaccines. Two mRNA vaccines were designed against high-risk type HPVs (HPV 16 and HPV 18) targeting the E6 and E7 oncoproteins. Here, we utilized advanced immunoinformatics approaches to predict potential epitopes, including helper T lymphocyte (HTL), cytotoxic T lymphocyte (CTL), and B-cell epitopes derived from the E6 and E7 oncoproteins. After being assessed for antigenicity, allergenicity, and toxicity, the final vaccine was constructed using highly prioritized epitopes. Further physicochemical profiling, structural prediction, validation, molecular docking, simulations, *in silico* cloning, and immune simulations were performed to evaluate the vaccine’s stability, functionality, and suitability.

## Methods

### Sequence retrieval

All available amino acid sequences of the E6 and E7 proteins of HPV 16 and HPV 18 were retrieved from the National Center for Biotechnology Information (NCBI) (https://www.ncbi.nlm.nih.gov/) protein database in FASTA format [58]. The protein sequences were then aligned with MEGA X software to generate a consensus sequence. The consensus sequences of the proteins E6 and E7 were then applied for subsequent vaccine construction.

### Helper T lymphocyte (HTL) binding epitope prediction

HTL binding or histocompatibility complex-I (MHC-I) epitopes of the selected proteins (E6 and E7) were predicted by the Immune Epitope Database (IEDB) [59, 60] and Net-MHC 4.0 (http://www.cbs.dtu.dk/services/NetMHC/) [61, 62] server. The IEDB is a comprehensive database that contains information on antibodies, B- and T-cell epitopes, MHC molecules, and MHC binding ligands in humans and animal species, including primates and mice [59, 62–74]. HTL epitope binding was forecasted with the IEDB’s recommended NetMHCpan 4.1 EL prediction method, utilizing a low percentile rank (<1.00) as the selection criteria. A lower percentile score indicates more affinity for the epitopes [75, 76]. The human allele reference sets were used to predict HTL binding. By analyzing ligand data and MHC-I binding affinities, the NetMHC 4.0 server can foretell how MHC-I will interact with peptides [59, 61, 73]. The server’s default parameter was employed in subsequent HTL epitope prediction. Finally, the selected epitopes were screened for physiological features including antigenicity, allergenicity, and toxicity by VaxiJen 2.0 (http://www.ddg-pharmfac.net/vaxijen/VaxiJen/VaxiJen.html) [77], AllerTOP v. 2.0 (https://www.ddg-pharmfac.net/AllerTOP/index.html) [78] and ToxinPred (https://webs.iiitd.edu.in/raghava/toxinpred/algo.php) [79] server, respectively. All parameters relating to the servers were left in their default settings.

The article "Designing of an mRNA vaccine against high-risk human papillomavirus targeting the E6 and E7 oncoproteins exploiting immunoinformatics and dynamic simulation" was retracted in 2025. Reasons: compromised peer review; unreliable results or conclusions.

### Cytotoxic T lymphocyte (CTL) binding epitope prediction

CTL binding or histocompatibility complex-II (MHC-II) epitopes of the selected proteins (E6 and E7) were predicted using the IEDB [59, 60] and NetMHCIIpan 4.0 server (http://www.cbs.dtu.dk/services/NetMHCIIpan/) [60, 80]. CTL epitope binding was predicted via the IEDB’s NetMHCIIpan 4.1 EL prediction method, employing a low percentile rank cutoff (<1.00), with human allele reference sets used for CTL binding prediction [75, 76, 81]. The NetMHCIIpan 4.0 server (http://www.cbs.dtu.dk/services/NetMHCIIpan/) utilizes the Artificial Neural Networks (ANNs) for the MHC-II binding epitope prediction [60, 80]. The default parameter of the server was utilized in the prediction of CTL epitopes. Following epitope selection, the epitopes were further assessed for antigenicity, allergenicity, and toxicity by VaxiJen 2.0 [77], AllerTOP v. 2.0 [78], and ToxinPred server, respectively [79]. Finally, the epitopes were assessed for interferon-gamma (IFN-γ) induction by the IFNepitope server (https://webs.iiitd.edu.in/raghava/ifnepitope/design.php). We used the IFNepitope server’s Design Module and Hybrid (Motif + SVM) prediction technique to determine whether the expected HTL epitopes might induce IFN-gamma [75, 76]. The epitopes that passed all the parameters were then proceeded for the vaccine construction.

### Linear B-cell epitope prediction

The linear B-cell epitopes of the protein of interest (E6 and E7) were predicted by the IEDB and the ABCpred (https://webs.iiitd.edu.in/raghava/abcpred/ABC_submission.html) server [82]. The IEDB server uses Hidden Markov Model (HMM) approach to estimate linear B-cell epitopes based on the sequence properties of the antigen [83]. Conversely, the ABCpred server utilizes an HMM and a propensity scale approach to compute the linear B-cell epitopes [82]. During the prediction, all the parameters were kept as default respective to the servers. The selected epitopes were, therefore, screened for antigenic, allergenic, and toxigenic characteristics by VaxiJen 2.0 [77], AllerTOP v. 2.0 [78], and ToxinPred server, respectively [79].

The article "Designing of an mRNA vaccine against high-risk human papillomavirus targeting the E6 and E7 oncoproteins exploiting immunoinformatics and dynamic simulation" was retracted in 2025. Reasons: compromised peer review; unreliable results or conclusions.

### Vaccine mapping

The mapping of vaccine 1 (V1) and vaccine 2 (V2) was carried out by using the highly prioritized epitopes of the selected proteins (E6 and E7). As an immune stimulant, the adjuvants, heparin-binding hemagglutinin (HBHA) and 50S ribosomal protein L7/L12, were used in the V1 and V2, respectively. Suitable linkers, including EAAAK, AYY, AK, and KFER, were used in the final vaccine mapping [53, 84, 85]. These linkers facilitate the vaccine components’ proper folding, stability, and flexibility, augmenting the immunological response [86–88].

### Evaluation of physicochemical properties

The physicochemical properties of the V1 and V2, including the molecular weight, the total number of amino acids, instability, aliphatic index, isoelectric point (pI), grand average of hydropathicity (GRAVY), the total number of positively and negatively charged residues, and the total number of atoms, were predicted by Expasy’s ProtParam server (http://web.expasy.org/protparam/) [89]. Following that, the solubility of the V1 and V2 was predicted by the SOLpro (https://scratch.proteomics.ics.uci.edu/) and SOSUI server (https://harrier.nagahama-i-bio.ac.jp/sosui/mobile/) [90–93]. The probable allergenic reactions of the V1 and V2 were assessed by AllergenFP v.1.0 (http://ddg-pharmfac.net/AllergenFP/), AllerCatPro v.2.0 (https://allercatpro.bii.a-star.edu.sg/) [94] and AlgPred (https://webs.iiitd.edu.in/raghava/algpred/submission.html) server. The antigenic features of the vaccines were also estimated by ANTIGENpro (http://scratch.proteomics.ics.uci.edu) [95] and VaxiJen 2.0 (http://www.ddg-pharmfac.net/vaxijen/VaxiJen/VaxiJen.html) server [77]. The threshold value was set up for this analysis using the default setting of 0.5.

### Secondary structure prediction

The secondary structures of the V1 and V2 were predicted by the GOR4 (https://npsa-prabi.ibcp.fr/cgi-bin/npsa_automat.pl?page=/NPSA/npsa_gor4.html), SOPMA (https://npsa-prabi.ibcp.fr/cgi-bin/npsa_automat.pl?page=/NPSA/npsa_sopma.html) and PSIPRED (http://bioinf.cs.ucl.ac.uk/psipred/) [96–99]. While predicting the secondary structure, the GOR4 utilizes information theory and Bayesian statistics [100]. The SOPMA, on the other hand, predicts a three-state illustration (alpha-helix, beta-sheet, and coil) of the secondary structure via a homology modeling approach [98]. Contrarily, the PSIPRED server utilizes two feed-forward neural networks and PSI-BLAST (protein-specific iterated basic local alignment search tool) to predict the secondary structure [101].

### Tertiary structure prediction, refinement, and validation

The tertiary structures (3D) of the V1 and V2 were predicted by the I-TASSER server (https://zhanggroup.org/I-TASSER/). The server performs multiple threading alignments and iterative template fragment assembly simulations to predict the 3D structure of a protein [74, 102]. The 3D structures of the vaccines were applied for further structural refinement by the GalaxyWEB server [103]. Further structural validations of the V1 and V2 were carried out by the SAVES v6.0 server (https://saves.mbi.ucla.edu/), which defines the stereochemical quality of the predicted vaccine models through Ramachandran plot and ERRAT analysis [104–108]. Finally, we utilized the ProSA-web server (https://prosa.services.came.sbg.ac.at/prosa.php) to assess the structural accuracy of the predicted 3D model structure. The server provides a Z-score for a predicted 3D model structure, indicating the correctness and probable flaws of the model [57, 76, 109].

The article "Designing of an mRNA vaccine against high-risk human papillomavirus targeting the E6 and E7 oncoproteins exploiting immunoinformatics and dynamic simulation" was retracted in 2025. Reasons: compromised peer review; unreliable results or conclusions.

### Prediction of discontinuous B-cell epitopes

The discontinuous B-cell epitopes of the V1 and V2 were predicted by the DiscoTope 2.0 (http://www.cbs.dtu.dk/services/DiscoTope/) [110] and Ellipro (http://tools.iedb.org/ellipro/) server [111]. The DiscoTope 2.0 server performs through the surface accessibility computation [110], where the ElliPro server (http://tools.iedb.org/ellipro/) utilizes a combination of three algorithms during discontinuous B-cell epitope prediction [111].

### Disulfide engineering of the vaccines

Disulfide engineering is a technique used to introduce disulfide bonds within protein structures, enhancing their stability. These disulfide bonds strengthen the protein’s folded structure by reducing conformational entropy and increasing the free energy of the denatured state [112]. In this study, the Disulfide by Design 2.13 server (http://cptweb.cpt.wayne.edu/DbD2/) was employed to identify specific residue pairs within the vaccine construct that could potentially be mutated to cysteine, facilitating the formation of disulfide bonds. This strategic mutation can further stabilize the overall protein structure [113]. The server’s algorithm utilizes a geometric model based on native disulfide bonds to accurately calculate the χ3 torsion angle, using the 5th Cβ-Cβ distance as a reference. Given the variability in native disulfide bonds, the DbD2 server allows some flexibility in the Caf-Cβ-Sγ angle. DbD2 generates an estimated energy value for each potential disulfide bond, aiding in the ranking of candidates. Additionally, mutant PDB files can be produced for selected disulfide bonds for further analysis [76, 114].

### Molecular docking analysis

Before molecular docking analysis, the 3D structure of human toll-like receptor-2 (TLR-2) (PDB: 2Z7X) and toll-like receptor-4 (TLR-4) (PDB: 3FXI) were retrieved from the PDB (Protein data bank) database (www.rcsb.org) [115]. Subsequently, the docking analysis of vaccine—TLR-2 (V1—TLR-2 and V2—TLR-2) and vaccine—TLR-4 (V1—TLR-4 and V2—TLR-4) were carried out by the ClusPro 2.0 (cluspro.bu.edu/login.php) server [116–119]. The ClusPro 2.0 server operates through a series of three continuous phases: first, it performs rigid body docking; next, it clusters the lowest energy structures; and finally, it refines the structures through energy minimization [76, 118]. The complex with the lowest energy score and highest docking efficiency was selected as the best-docked candidate. The docked complexes were further visualized and analyzed by the PyMOL and PDBsum (http://www.ebi.ac.uk/thornton-srv/databases/pdbsum/Generate.html) server [84, 120].

The article "Designing of an mRNA vaccine against high-risk human papillomavirus targeting the E6 and E7 oncoproteins exploiting immunoinformatics and dynamic simulation" was retracted in 2025. Reasons: compromised peer review; unreliable results or conclusions.

### Free energy calculation by molecular mechanics with generalized Born and surface area solvation (MM-GBSA)

The free energies associated with the vaccine and TLRs interactions (V1—TLR-2, V2—TLR-2, V1—TLR-4, and V2—TLR-4) were calculated by the MM-GBSA program of the HawkDock server [121–123]. The program utilizes molecular mechanics and the Generalised Born approaches to analyze intermolecular interactions, including van der Waals forces (VDW), electrostatic interactions (ELE), polar (GB), and non-polar (SA) components [121–123].

### Molecular dynamic simulation

The GROningen MAchine for Chemical Simulations (GROMACS) (version 2022.3) [124] software was utilized for the molecular dynamic simulations of the vaccine and TLRs (V1—TLR-2, V1—TLR-4, V2—TLR-2 and V2—TLR-4) complexes along with the vaccine apo structures (V1 and V2). The GROMOS96 43a1 force field was applied for the simulation, where a cubic water box was built with an SPC water model. However, the system was neutralized using the NaCl. Finally, 100 nanoseconds (ns) molecular dynamic simulation was run using the equilibration type of isothermal-isochoric (NVT) and isobaric (NPT), temperature (K) of 300, pressure (bar) of 1.0, and a periodic boundary conditions and time integration step of 2 femtoseconds (fs). The trajectory data were analyzed at 100 picoseconds (ps) in the snapshot interval. After the successful simulation run, the root mean square deviation (RMSD), root mean square fluctuation (RMSF), radius of gyration (Rg), solvent accessible surface area (SASA), and hydrogen bond (H-bond) analysis were performed by the respective modules integrated within the GROMACS software.

### Codon optimization and *in silico* cloning

Codon optimization of the vaccines was performed by the Java Codon Adaptation Tool (JCat) server (http://www.jcat.de/Start.jsp) utilizing a bacterial expression system, *E*. *coli* strain K12. The server evaluates the expression level of the vaccines through codon adaptation index (CAI) and GC contents. However, the CAI value ≥ 0.8 is considered a good score, while the best score should be ≥ 1.0, and the GC contents, ranging from 30 to 70%, are acceptable [125, 126]. The optimized gene sequences of the vaccines were cloned in *E*. *coli* plasmid vector pET-28a(+) using EcoRI, BamHI, and NdeI restriction sites. Finally, the optimized sequences of the vaccines were inserted into the plasmid vector pET-28a(+) using the SnapGene software.

The article "Designing of an mRNA vaccine against high-risk human papillomavirus targeting the E6 and E7 oncoproteins exploiting immunoinformatics and dynamic simulation" was retracted in 2025. Reasons: compromised peer review; unreliable results or conclusions.

### Immune simulation

Using the C-ImmSim server, the immune simulations of the V1 and V2 were evaluated and predicted (https://kraken.iac.rm.cnr.it/C-IMMSIM/) [127]. The server uses a position-specific scoring matrix (PSSM) to predict a vaccine-mediated humoral and cellular immune response of a mammalian immune system [126, 128]. For proper immunization, the V1 and V2 were designed with three doses of the regime, which will be given at four-week intervals. The simulation run was carried out by the default parameters of the server, while the time steps were adjusted at 1 (day 1), 84 (day 28), and 168 (day 56) (a single step is equivalent to 8 hours of daily life) [85]. The recommended interval between two successive doses of most commercial immunizations is four weeks; thus, three shots must be delivered four weeks apart [76, 129]. Finally, the simulation volume was set to 50 with 1000 times the simulation steps. However, the random seed was chosen as the server’s default setting without adjoining lipopolysaccharides (LPS).

### mRNA structure prediction

The secondary structures of both the V1 and V2 vaccines were predicted by the RNAfold (http://rna.tbi.univie.ac.at/cgi-bin/RNAWebSuite/RNAfold.cgi) server [130]. During the prediction, the server provided thermodynamically derived minimum free energy (MFE) of the query mRNA structures [131, 132]. Before this analysis, the JCat optimized gene sequences (V1 and V2) were first transcribed into RNA sequences through the process of DNA>RNA conversion at http://biomodel.uah.es/en/lab/cybertory/analysis/trans.htm. Subsequently, these RNA sequences were applied to the RNAfold server for secondary structure prediction and validation.

## Results

### Sequence retrieval

After obtaining the protein sequences E6 and E7 of HPV 16 and HPV 18 from the NCBI database, the multiple sequence analysis (MSA) analysis provided two consensus FASTA sequences of the proteins. These consensus sequences were then applied for the subsequent vaccine development. Fig 1 illustrates an empirical overview of the entire vaccine design process.

The article "Designing of an mRNA vaccine against high-risk human papillomavirus targeting the E6 and E7 oncoproteins exploiting immunoinformatics and dynamic simulation" was retracted in 2025. Reasons: compromised peer review; unreliable results or conclusions.

**Fig 1:** The overview of the mRNA vaccine design against human papillomavirus 16 and human papillomavirus 18 targeting the E6 and E7 proteins.

### HTL binding epitope prediction

Both the IEDB and Net-MHC 4.0 server predicted several HTL peptides from which a total of twelve 9-mer length peptides were selected based on their affinity score and percentile rank (≤1.00) (Table 1). These peptide sequences were also predicted to be antigenic, non-allergic, and non-toxic and were applied for subsequent vaccine construction.

**Table 1:** List of selected HTL epitopes and their antigenicity, allergenicity, and toxicity.

Protein	Strain	Peptide	Alleles	Antigenicity	Allergenicity	Toxicity
E6	HPV 16	DPQERPRKL	HLA-A*01:01, HLA-A*03:01, HLA-A*23:01, HLA-A*30:01, HLA-A*30:02, HLA-A*31:01, HLA-A*33:01, HLA-B*07:02, HLA-B*08:01, HLA-B*15:01, HLA-B*35:01, HLA-B*51:01, HLA-B*53:01, HLA-B*57:01, HLA-B*58:01	Probable antigen (0.5782)	Probable non-allergen	Non-toxin (-1.27)
		CPEEKQRHL	HLA-A*01:01, HLA-A*02:01, HLA-A*03:01, HLA-A*23:01, HLA-A*26:01, HLA-B*07:02, HLA-B*08:01, HLA-B*15:01, HLA-B*35:01, HLA-B*51:01, HLA-B*53:01, HLA-B*57:01, HLA-B*58:01	Probable antigen (1.3689)	Probable non-allergen	Non-toxin (-0.82)
	HPV 18	VYCKTVLEL	HLA-A*01:01, HLA-A*03:01, HLA-A*23:01, HLA-A*24:02, HLA-A*26:01, HLA-A*30:01, HLA-A*30:02, HLA-A*31:01, HLA-A*32:01, HLA-A*33:01, HLA-B*07:02, HLA-B*08:01, HLA-B*15:01, HLA-B*35:01, HLA-B*51:01, HLA-B*53:01, HLA-B*57:01, HLA-B*58:01	Probable antigen (0.6120)	Probable non-allergen	Non-toxin (-0.92)
		RFHNIAGHY	HLA-A*01:01, HLA-A*02:01, HLA-A*02:03, HLA-A*03:01, HLA-A*23:01, HLA-A*24:02, HLA-A*26:01, HLA-A*30:01, HLA-A*30:02 HLA-A*31:01, HLA-A*32:01, HLA-A*33:01, HLA-B*07:02, HLA-B*08:01, HLA-B*15:01, HLA-B*35:01, HLA-B*51:01, HLA-B*53:01, HLA-B*57:01, HLA-B*58:01	Probable antigen (0.5004)	Probable non-allergen	Non-toxin (-0.66)
E7	HPV 16	RAHYNIVTF	HLA-A*01:01, HLA-A*02:01, HLA-A*02:03, HLA-A*03:01, HLA-A*23:01, HLA-A*24:02, HLA-A*26:01, HLA-A*30:01, HLA-A*30:02, HLA-A*31:01, HLA-A*32:01, HLA-A*33:01 HLA-B*07:02, HLA-B*08:01, HLA-B*15:01, HLA-B*35:01, HLA-B*51:01, HLA-B*53:01, HLA-B*57:01, HLA-B*58:01	Probable antigen (0.5919)	Probable non-allergen	Non-toxin (-1.05)
		LEDLLMGTL	HLA-A*01:01, HLA-A*02:01, HLA-A*02:03, HLA-A*03:01, HLA-A*23:01, HLA-A*24:02, HLA-A*26:01, HLA-A*30:01, HLA-A*30:02 HLA-A*31:01, HLA-A*32:01, HLA-A*33:01, HLA-B*07:02, HLA-B*15:01, HLA-B*35:01 HLA-B*57:01, HLA-B*58:01	Probable antigen (0.8392)	Probable non-allergen	Non-toxin (-1.19)
	HPV 18	KTLSFVCPW	HLA-A*01:01, HLA-A*02:01, HLA-A*02:03, HLA-A*03:01, HLA-A*23:01, HLA-A*24:02, HLA-A*26:01, HLA-A*30:01, HLA-A*30:02, HLA-A*31:01, HLA-A*32:01, HLA-A*33:01, HLA-B*07:02, HLA-B*08:01, HLA-B*15:01, HLA-B*35:01, HLA-B*51:01, HLA-B*53:01, HLA-B*57:01, HLA-B*58:01	Probable antigen (1.3290	Probable non-allergen	Non-toxin (-0.50)
		EIDGVNHQH	HLA-A*01:01, HLA-A*02:01, HLA-A*03:01, HLA-A*30:01, HLA-A*30:02, HLA-A*31:01, HLA-B*07:02, HLA-B*08:01, HLA-B*15:01, HLA-B*35:01, HLA-B*51:01, HLA-B*53:01, HLA-B*57:01, HLA-B*58:01	Probable antigen (0.9980)	Probable non-allergen	Non-toxin (-0.92)

The article "Designing of an mRNA vaccine against high-risk human papillomavirus targeting the E6 and E7 oncoproteins exploiting immunoinformatics and dynamic simulation" was retracted in 2025. Reasons: compromised peer review; unreliable results or conclusions.

### CTL binding epitope prediction

The CTL binding epitopes of the selected proteins, the E6 and E7 proteins of HPV 16 and HPV 18, were predicted by the IEDB and NetMHCIIpan 4.0 server. Based on affinity and percentile score, twelve 15-mer length peptides were selected. The selected peptide sequences were also reported to have antigenic, non-allergenic, and non-toxic properties. No IL-10-producing capabilities of the selected epitopes were found, but these have IFN-γ inducing capabilities (Table 2).

**Table 2:** List of selected CTL epitopes with their antigenicity, allergenicity, IFN-γ and IL-10 inducing capability, and toxicity.

Proteins	Strain	Peptides	Alleles	Antigenicity	Allergenicity	IFN-γ	IL-10 prediction	Toxicity
E6	HPV 16	QQLLRREVYDFAFRD	HLA-DRB1*03:01, HLA-DRB1*07:01, HLA-DRB1*15:01, HLA-DRB3*01:01, HLA-DRB3*02:02, HLA-DRB4*01:01, HLA-DRB5*01:01	Probable antigen (0.5512)	Probable non-allergen	Positive	IL10 non-inducer	Non-toxin
		KKQRFHNIRGRWTGR	HLA-DRB1*03:01, HLA-DRB1*07:01, HLA-DRB1*15:01, HLA-DRB3*01:01, HLA-DRB3*02:02, HLA-DRB4*01:01, HLA-DRB5*01:01	Probable antigen (1.0979)	Probable non-allergen	Positive	IL10 non-inducer	Non-toxin
	HPV 18	EKRRFHNIAGHYRGQ	HLA-DRB1*03:01, HLA-DRB1*07:01, HLA-DRB1*15:01, HLA-DRB3*01:01, HLA-DRB3*02:02, HLA-DRB4*01:01, HLA-DRB5*01:01	Probable antigen (0.6494)	Probable non-allergen	Positive	IL10 non-inducer	Non-toxin
		LNEKRRFHNIAGHYR	HLA-DRB1*03:01, HLA-DRB1*07:01, HLA-DRB1*15:01, HLA-DRB3*01:01, HLA-DRB3*02:02, HLA-DRB4*01:01, HLA-DRB5*01:01	Probable antigen (0.8789)	Probable non-allergen	Positive	IL10 non-inducer	Non-toxin
E7	HPV 16	TLHEYMLDLQPETTD	HLA-DRB1*03:01, HLA-DRB1*07:01, HLA-DRB1*15:01, HLA-DRB3*01:01, HLA-DRB3*02:02, HLA-DRB4*01:01, HLA-DRB5*01:01	Probable antigen (1.0256)	Probable non-allergen	Positive	IL10 non-inducer	Non-toxin
		CVQSTHVDIRTLEDL	HLA-DRB1*03:01, HLA-DRB1*07:01, HLA-DRB1*15:01, HLA-DRB3*01:01, HLA-DRB3*02:02, HLA-DRB4*01:01, HLA-DRB5*01:01	Probable antigen (1.0262)	Probable non-allergen	Positive	IL10 non-inducer	Non-toxin
	HPV 18	IDGVNHQHLPARRAE	HLA-DRB1*03:01, HLA-DRB1*07:01, HLA-DRB1*15:01, HLA-DRB3*01:01, HLA-DRB3*02:02, HLA-DRB4*01:01, HLA-DRB5*01:01	Probable antigen (0.7585)	Probable non-allergen	Positive	IL10 non-inducer	Non-toxin
		EIDGVNHQHLPARRA	HLA-DRB1*03:01, HLA-DRB1*07:01, HLA-DRB1*15:01, HLA-DRB3*01:01, HLA-DRB3*02:02, HLA-DRB4*01:01, HLA-DRB5*01:01	Probable antigen (0.6718)	Probable non-allergen	Positive	IL10 non-inducer	Non-toxin

The article "Designing of an mRNA vaccine against high-risk human papillomavirus targeting the E6 and E7 oncoproteins exploiting immunoinformatics and dynamic simulation" was retracted in 2025. Reasons: compromised peer review; unreliable results or conclusions.

### Linear B-cell epitope prediction

The linear B-cells of the selected proteins, the E6 and E7 proteins of HPV 16 and HPV 18, were predicted by the IEDB and the ABCpred servers. Twelve 16-mer epitopes were selected that have no toxic and allergenic properties but show antigenic properties (Table 3).

**Table 3:** List of selected linear B-cell epitopes with their toxicity, allergenicity, and antigenicity.

Proteins	Strains	Peptides	Toxicity	Allergenicity	Antigenicity
E6	HPV 16	ERPRKLPQLCTELQTT	Non-toxin	Probable non-allergen	Probable antigen (0.6858)
		QTTIHDIILECVYCKQ	Non-toxin	Probable non-allergen	Probable antigen (0.4560)
		TRRPYKLPDLCTELNT	Non-toxin	Probable allergen	Probable antigen (0.6763)
		LQDIEITCVYCKTVLE	Non-toxin	Probable non-allergen	Probable antigen (1.3738)
E7	HPV 18	LQPETTDLYCYEQLND	Non-toxin	Probable non-allergen	Probable antigen (1.0269)
		DGPAGQAEPDRAHYNI	Non-toxin	Probable non-allergen	Probable antigen (0.5342)
		KATLQDIVLHLEPQNE	Non-toxin	Probable non-allergen	Probable antigen (1.0940)
		SDSEEENDEIDGVNHQ	Non-toxin	Probable non-allergen	Probable antigen (0.6299)

### Vaccine mapping

The selected epitopes of the proteins E6 and E7 were used in the final vaccine mapping (Tables 1–3). Two different vaccine candidates were mapped using the selected epitopes, adjuvants, and linkers. The adjuvant, HBHA was connected to the V1 with the EAAK linker, while the HTL, CTL, and linear B-cell epitopes were connected with each other by AYY, AK, and KFER linkers, respectively (Fig 2A). For the V2, 50S ribosomal protein L7/L12 adjuvant was connected with the EAAK linker, while the rest of the epitopes, including the HTL, CTL, and linear B-cell epitopes, were connected by AYY, AK, and KFER linkers, respectively (Fig 2B).

**Fig 2:** The designed vaccine candidates V1 (A) and V2 (B) against HPV 16 and HPV 18. The schematic presentation of the vaccines containing adjuvant (yellow color), epitopes (MHC-I-green, MHC-II- transparent orange, linear B-cell-light blue), and linkers (EAAAK- deep blue, AYY-light blue, AK-purple, and KFER-maroon).

### Evaluation of physicochemical properties

The physicochemical properties of the V1 and V2 were obtained from the ExPASy ProtPram server. According to the server, V1 constituted a total number of 592 amino acids, while V2 constituted 523 amino acids. The molecular weight of the V1 and V2 were predicted to be 68551.58 Da and 60457.60 Da, respectively. The V1 has been reported as basic in nature, with an isoelectric point (pI) of 8.73, while V2 has been reported as acidic in nature, with a pI score of 6.62. The GRAVY of the V1 and V2 were predicted to be -0.811 and -0.648, respectively, indicating that both vaccines were predicted to be water-soluble (hydrophilic). The aliphatic index of the V1 was predicted to be 84.33, whereas it was predicted to be 78.26 for the V2. Both the vaccines, V1 and V2, were predicted to be unstable, with instability indices of 61.89 and 57.24, respectively (Table 4). Additionally, both the V1 and V2 vaccines were predicted to be water soluble, non-allergenic, and antigenic proteins (Table 4).

The article "Designing of an mRNA vaccine against high-risk human papillomavirus targeting the E6 and E7 oncoproteins exploiting immunoinformatics and dynamic simulation" was retracted in 2025. Reasons: compromised peer review; unreliable results or conclusions.

**Table 4:** The physicochemical and immunological properties of the V1 and V2.

Physicochemical properties	V1	V2
Molecular Weight (Da)	68551.58	60457.60
Number of amino acids	592	523
Theoretical pI	8.73	6.62
GRAVY	-0.811	-0.648
Aliphatic index	84.33	78.26
Instability index	61.89	57.24
Total number of negatively charged residues (Asp+Glu)	91	84
Total number of positively charged residues (Arg+Lys)	100	80
Solubility (SOSUI/SOLpro)	Soluble protein	Soluble protein
Allergenicity (AllergenFP v.1.0/ AllerCatPro v.2.0/ AlgPred)	Probable non-allergen	Probable non-allergen
Antigenicity (ANTIGENpro/VaxiJen 2.0)	Probable antigen	Probable antigen

### Secondary structure prediction

Utilizing the three distinct servers (GOR4, SOPMA, and PSIPRED), the secondary structures of the vaccines (V1 and V2) were predicted and evaluated. The GOR4 server predicted 29.73% random coil, 61.15% alpha helix, and 9.12% extended strands (beta sheet) in V1; in comparison, the SOPMA server predicted random coil of 27.03%, an alpha helix of 66.05%, and extended strands of 6.93% (S1 Fig). For V2, the GOR4 server indicated that the secondary structure of the V2 has 35.76% random coil, 51.83% alpha helix, and 12.43% extended strands (beta sheet), while the SOPMA predicted 32,70% random coil, 57.93% alpha helix and 9.37% extended strands (S1 Fig). Additionally, the PSIPRED server provided the features of the vaccines’ secondary structure through three-state prediction (coil, helix, and strands) (Fig 3, S2 Fig).

**Fig 3:** The secondary structure of the V1 (A) and V2 (B) predicted by PSIPRED. A larger bar indicates a higher confidence level, and the first bar (Conf) represents that degree of confidence in the forecast. In the second bar (Cart), the vaccine’s beta-sheet, helix, and coil structures are yellow, pink, and grey, respectively. The third bar (Pred) represents a structural feature, and the fourth bar (AA) represents an amino acid sequence.

### Tertiary structure prediction, refinement, and validation

For the V1, out of the five models predicted by the I-TASSER server, the model with the greatest C-score of -0.86, TM-score of 0.51±0.15, and RMSD of 11.7±4.5Å was chosen for further investigation; in contrast, the V2 model with the greatest C-score of -0.61, TM-score of 0.64±0.13, and RMSD of 8.8±4.6Å was chosen. Subsequently, both the predicted models were then applied for structural refinement by the GalaxyWEB server. The refined 3D model of the V1 was given RMSD, MolProbity score, and Ramachandran’s favored region of 0.410, 1.674, and 97.3%, respectively. On the other hand, the refined 3D model of the V2 was found with RMSD, MolProbity score, and Ramachandran’s favored region of 0.525, 2.205, and 92.1%, respectively. These findings indicated that both proteins have well-stable 3D structures. According to the Ramachandran plot analysis, the V1 model had 94.5% amino acid residues in the most favored region, 4.2% in the additional allowed region, and 0.5% in the generously allowed region (Fig 4A). At the same time, the V2 had 87.1% amino acid residues in the most favored region, 9.6% in the additional allowed region, and 0.6% in the generously allowed region (Fig 4A). The Z score of the V1 and V2 were predicted to be -5.15 and -4.1, respectively (Fig 4B). Also, the ERRAT scores for the refined V1 and V2 were calculated as 92.771 and 83.497, respectively (Fig 4D).

The article "Designing of an mRNA vaccine against high-risk human papillomavirus targeting the E6 and E7 oncoproteins exploiting immunoinformatics and dynamic simulation" was retracted in 2025. Reasons: compromised peer review; unreliable results or conclusions.

**Fig 4:** Validation of the I-TASSER predicted models of the vaccines (V1 and V2). The refined 3D structures are evaluated through the Ramachandran plot (A), Z score (B), and ERRAT (D).

### Prediction of discontinuous B-cell epitopes

The DiscoTope 2.0 server identified 290 and 252 discontinuous B-cell epitope residues in the V1 and V2 structures, respectively (Fig 5 and S1 Table). In the case of V1, the epitopes have different scoring ranges from 0.524 to 0.86 with an individual number of residues, whereas the epitopes from V2 have different scoring ranges from 0.519 to 0.79 (S1 Table).

**Fig 5:** The discontinuous B-cell epitopes of the V1 (A) and V2 (B) were predicted by DiscoTope 2.0. The discontinuous B-cell epitopes were illustrated as yellow-color surfaces, while the whole vaccine portions were displayed with grey sticks.

### Disulfide engineering of the vaccines

Through disulfide engineering, it was discovered that V1 included 20 pairs of amino acid residues, but V2 contained 31 pairs of residues capable of establishing disulfide bonds. Between -87 and +97 degrees, χ3 peaks in 1505 native disulfide linkages in 331 non-homologous proteins were observed, with 90% of spontaneously produced bonds having an energy value below 2.2 kcal/mol [113]. Following the scrutiny of the χ3 and B-factor characteristics of the residue pairs based on energy, two pairs were chosen for V1 (LYS 178- TYR 418, ALA 201-HIS 390, and GLY 244- ALA 344), while three pairs were chosen for V2 (GLY 46-ASP 98, GLY 89-ASP 136, and LEU 188- ALA 200) (S3 Fig). With the addition of cysteine, these pairings were altered.

The article "Designing of an mRNA vaccine against high-risk human papillomavirus targeting the E6 and E7 oncoproteins exploiting immunoinformatics and dynamic simulation" was retracted in 2025. Reasons: compromised peer review; unreliable results or conclusions.

### Molecular docking study

The docking analysis of the vaccines and human receptors (TLR-2 and TLR-4) was performed by the ClusPro 2.0 server. The server has generated 30 models for each complex, from which the models having the lowest energy scores of -1159.3, -1109.3, -1246.3, and -1244.8 were chosen for the “V1—TLR-2”, “V1—TLR-4”, “V2—TLR-2” and the “V2—TLR-4”, respectively (Fig 6; Table 5). Additionally, the center energy scores of the “V1—TLR-2”, “V1—TLR-4”, “V2—TLR-2” and “V2—TLR-4” were found to be -1159.3, -1109.3, -1140.8 and -1244.8, respectively (Fig 6; Table 5). However, the docked vaccine-TLRs complexes were visualized and analyzed by PyMOL and PDBsum. According to PDBsum, the “V1—TLR-2” complex has nine hydrogen bonds, 25 salt bridges, and 235 non-bond interactions (Fig 6A; Table 5), whereas the “V1—TLR-4” complex has 7 hydrogen bonds, 23 salt bridges and 224 non-bond interactions (Fig 6B; Table 5). Additionally, the “V2—TLR-2” complex has 8 hydrogen bonds, 17 salt bridges, and 231 non-bond interactions (Fig 6C; Table 5), whereas the “V2—TLR-4” complex has 7 hydrogen bonds, 38 salt bridges, and 421 non-bond interactions (Fig 6D; Table 5).

**Fig 6:** The interaction between “V1—TLR-2” (A), “V1—TLR-4” (B), “V2—TLR-2” (C), and “V2—TLR-4” (D) complexes. The vaccines V1 and V2 and the receptors TLR-2 and TLR-4 are depicted as green, red, cyan, and purple, respectively. At the same time, their interactions are denoted with multiple colors, following the characteristics of the bonds.

**Table 5:** The docking scores and inter-molecular interactions between the vaccine-TLRs complexes.

Vaccine	Complex	Weighted Score		Interactions between the vaccine and TLRs			
		Center	Lowest energy	Salt bridges	Disulphide bonds	Hydrogen bonds	Non-bonded contacts
V1	Vaccine-TLR-2	-1159.3	-1159.3	9	-	25	235
	Vaccine-TLR-4	-1109.3	-1109.3	7	-	23	224
V2	Vaccine-TLR-2	-1140.8	-1246.3	8	-	17	231
	Vaccine-TLR-4	-1244.8	-1244.8	7	-	38	421

### Free energy calculation by MM-GBSA

For the MM-GBSA analysis, we utilized the HawkDock server. This analysis revealed that the “V1—TLR-2” complex has the VDW, ELE, GB, and SA scores of -221.68, -1718.59, 1815.14, and -30.17 kcal/mol, respectively, and a total binding free energy of -155.29 (kcal/mol) (S3 Fig). Regarding the “V1—TLR-4” complex, the VDW, ELE, GB, and SA were calculated to be -186.44, -1068.74, 1182.46, and -23 kcal/mol, respectively with the total binding free energy of -95.72 kcal/mol (S4 Fig). On the other hand, the calculated MM-GBSA values for the "V2—TLR-2" complex was predicted to be -230.59 kcal/mol for VDW, -571.77 kcal/mol for ELE, 758.29 kcal/mol for GB, and -28.91 kcal/mol for SA. Following that, the complex was also reported with a total binding free energy of -72.97 kcal/mol (S4 Fig). Additionally, the V2—TLR-4 complex was analyzed, and the following MM-GBSA values were obtained: -331.1 kcal/mol for VDW energy, -342.91 kcal/mol for ELE energy, 530.07 kcal/mol for GB energy, and -44.74 kcal/mol for SA energy. Nevertheless, the complex was found to have a high binding free energy of -188.68 kcal/mol (S4 Fig).

The article "Designing of an mRNA vaccine against high-risk human papillomavirus targeting the E6 and E7 oncoproteins exploiting immunoinformatics and dynamic simulation" was retracted in 2025. Reasons: compromised peer review; unreliable results or conclusions.

### Molecular dynamic simulation

#### RMSD analysis

The RMSD of the vaccines (V1 and V2) and vaccine-TLR complexes (V1—TLR-2, V1—TLR-4, V2—TLR-2, and V2—TLR-4) structures were calculated to evaluate the stability of these complexes. Throughout the 100ns run, the RMSD values for the V1 and V1—TLR-4 steadily increased, while the RMSD values for V1—TLR-2 were drastically improved. But the RMSD of these complexes tended to decrease after a 100ns simulation run (Fig 7A). At the halfway of the simulation run (50ns), the differences in RMSD values of these complexes were clearly evident, which remained at the end of the 100ns simulation run. After the 100ns run, the average RMSD values for V1, V1—TLR-2, and V1—TLR-4 were calculated to be 0.106 nm, 0.116 nm, and 0.081 nm, respectively. These findings indicated that the V1 obtained a more stable structure when bound to TLR-4 than TLR-2 (Fig 7A). The RMSD values for the V2 and V2—TLR-2 were steadily increased, while the RMSD values for V2—TLR-2 showed a fluctuated plot; however, values started to decrease again after the 100 ns simulation run (Fig 7A). At the end of the complete simulation run, the average RMSD values for V2, V2—TLR-2, and V2—TLR-4 were calculated to be 0.737 nm, 0.738 nm, and 0.860 nm, respectively. Therefore, V2 was stable enough to be bound to TLR-2 rather than TLR-4 (Fig 7A).

**Fig 7:** The root mean square deviation (RMSD) (A), root mean square fluctuation (RMSF) (B), radius of gyration (Rg) (C), and solvent accessible surface area (SASA) (D) analyses of the vaccines (V1 and V2) and vaccine-TLR structures.

#### RMSF analysis

Additionally, the RMSF of these complexes was used to assess regional flexibility. Throughout the simulation, the motility pattern of the V1—TLR-2 is significantly different than V1 and V1—TLR-4 (Fig 7B), especially at the C and N terminals. In its unbound state, the V1 residues exhibited an average RMSF value of 0.80 nm, indicating moderate flexibility. However, this dynamic behavior significantly changed when V1 interacted with TLRs. Upon binding to TLR-2, the average RMSF value of V1 decreased to 0.61 nm, suggesting that the interaction stabilized the V1 residues, reducing their flexibility. Similarly, when bound to TLR-4, the RMSF value was reported as 0.71 nm, again reflecting a reduction in flexibility compared to the unbound state, though to a lesser extent than with TLR-2. In the case of V2, the motility pattern of RMSF of the V2—TLR-4 was notably different from the V2 and V2-TLR-2 (Fig 7B). During the simulation, the V2 domain showed distinct fluctuation patterns depending on whether it was bound to TLR-2 or TLR-4. The residues of V2 bound to TLR-4 exhibited more abrupt and pronounced fluctuations, indicating significant flexibility and instability during the interaction. Conversely, in both the unbound state and when bound to TLR-2, the V2 residues maintained more steady fluctuations. At the end of the 100ns simulation run, the average RMSF values for V2 were measured. For the unbound, the average RMSF was 0.29 nm, reflecting moderate flexibility. When bound to TLR-2, the RMSF decreased to 0.25 nm, suggesting that the interaction stabilized the V2 residues and reduced their movement. In contrast, the binding of V2 to TLR-4 resulted in a significantly higher RMSF value of 0.56 nm, indicating increased fluctuation and flexibility (Fig 7B).

The article "Designing of an mRNA vaccine against high-risk human papillomavirus targeting the E6 and E7 oncoproteins exploiting immunoinformatics and dynamic simulation" was retracted in 2025. Reasons: compromised peer review; unreliable results or conclusions.

#### Rg analysis

The Rg value of the V1—TLR-2 was higher than the Rg values of the V1 and V1—TLR-4 throughout the simulation run. Following the completion of the simulation, the Rg for the V1 was determined to be 2.96 nm. On the other hand, the Rg values obtained by the V1—TLR-2 and V1—TLR-4 complexes were 3.46 nm and 3.24 nm, respectively. Based on these findings, it can be inferred that the V1 exhibits a higher structural stability level when paired with TLR-4. Additionally, the Rg value of the V2—TLR-2 was higher than the Rg values of V2 and V2—TLR-4 (Fig 7C). After the simulation (100ns), the Rg for the V2 was measured as 2.96 nm, indicating the vaccine’s relatively compact structure in its unbound state. When V2 engaged with the TLR-2 and TLR-4, notable variations in Rg values were observed. The Rg value for the V2—TLR-2 complex spiked significantly to 3.79 nm, indicating a more expanded and less compact structure than the unbound V2. The V2—TLR-4 complex exhibited an Rg of 3.53 nm, suggesting a slightly more compact structure than V2—TLR-2, yet it remained more extended than the unbound V2 protein. The findings suggested that the interaction of V2 with various receptors affects its structural configuration, with TLR-2 causing a more significant structural expansion than TLR-4 (Fig 7C).

The article "Designing of an mRNA vaccine against high-risk human papillomavirus targeting the E6 and E7 oncoproteins exploiting immunoinformatics and dynamic simulation" was retracted in 2025. Reasons: compromised peer review; unreliable results or conclusions.

#### SASA analysis

After a 100ns simulation run, the SASA plot of the V1, V1—TLR-2, and V1—TLR-4 were almost identical throughout the simulation run. After the 100ns simulation, V1—TLR-2 had the highest SASA value out of V1 and V1—TLR-4. At the end of the simulation, an average SASA value of 261.55 nm^2^ was shown by the V1 itself. In contrast, the V1—TLR-2 and V1—TLR-4 complexes had significantly higher SASA values of 291.29 nm^2^ and 275.51 nm^2^, respectively. These findings demonstrated that the V1—TLR-2 complex was exposed to more solvent throughout the simulation, which could indicate that the V1 was more flexible or had a different shape when bound to TLR-2. While V1 singly was the most compact with the least solvent exposure, the intermediate SASA value of V1—TLR-4 showed a comparable but considerably less apparent impact (Fig 7D).

In the meantime, the SASA values of the V2 were consistently lower than those of its complexes with TLR-2 and TLR-4. The SASA quantifies the surface area of a biomolecule that is accessible to a solvent, frequently reflecting structural stability, folding, or possible interaction sites. During the simulation, the SASA values of the V2—TLR-2 and V2—TLR-4 complexes exhibited little variation, indicating no substantial difference in solvent exposure between the two complexes. A significant change occurred at the end of the complete simulation run. The V2—TLR-2 complex had the highest SASA value compared to the three configurations: V2 solely V2—TLR-2 and V2—TLR-4. The average SASA value of the V2 solely was 420.43 nm^2^, indicating a more compact or less solvent-exposed conformation. Nevertheless, the formation of complexes between V2 and TLR-2, as well as TLR-4, resulted in a significant elevation in the SASA values. The V2—TLR-2 complex exhibited an average SASA of 662.76 nm^2^, while the V2—TLR-4 complex had a lower, although still significant, SASA of 643.99 nm^2^ (Fig 7D). The augmentation in SASA for the complexes suggested that the V2 undergoes structural modifications upon interaction with TLR-2 and TLR-4, likely revealing a greater surface area to the surrounding solvent.

#### H-bond analysis

The simulation showed fluctuations in the number of hydrogen bonds in the docked complexes across different time intervals. At the beginning of the simulation (0 ns), the initial counts of hydrogen bonds were recorded as follows: V1—TLR-2 showed ten hydrogen bonds, V1—TLR-4 presented 11, V2—TLR-2 revealed 13, and V2—TLR-4 achieved a total of 16 hydrogen bonds. As the simulation progressed, significant changes were observed. At the 25 ns trajectory, the number of hydrogen bonds changed to 14 for V1—TLR-2, 16 for V1—TLR-4, 13 for V2—TLR-2, and a notable rise to 26 for V2—TLR-4. More alterations persisted during the simulation (S5 Fig). At the midpoint (50 ns), V1—TLR-2 showed an increase to 18 hydrogen bonds, whereas V1—TLR-4 stayed constant at 16. Conversely, V2—TLR-2 recognized a reduction to 12, while V2—TLR-4 significantly increased to 31 hydrogen bonds. At the end of a 100 ns simulation trajectory, the hydrogen bond analysis for two different ligand variations, V1 and V2, with TLR-2 and TLR-4 revealed notable patterns. The analysis showed that V1 formed 21 hydrogen bonds with TLR-2 and 13 hydrogen bonds with TLR-4. On the other hand, V2 demonstrated different binding characteristics, forming 15 hydrogen bonds with TLR-2 but a significantly higher number with TLR-4, recording 36 hydrogen bonds. (S5 Fig).

The article "Designing of an mRNA vaccine against high-risk human papillomavirus targeting the E6 and E7 oncoproteins exploiting immunoinformatics and dynamic simulation" was retracted in 2025. Reasons: compromised peer review; unreliable results or conclusions.

### Codon optimization and *in silico* cloning

The codon optimization of the V1 and V2 vaccines was facilitated by the Java Codon Adaptation Tool (JCat) using *E*. *coli* strain K12. The server predicted optimized codon sequences of 1776 and 1569 nucleotide length for V1 and V2, respectively (Fig 8). Besides, the adapted sequences’ codon optimization index (CAI) values were calculated as 1.0 for each vaccine. At the same time, the average GC content of the adapted V1 and V2 sequences were calculated as 51.88% and 51.63%, respectively. Finally, the adapted vaccine sequences were inserted into the plasmid vector pET-28a(+), SnapGene software to establish recombinant plasmid sequences (Fig 8).

**Fig 8:** *In silico* cloning of the pET-28a(+) plasmid vector with the inserts V1 (A) and V2 (B). SnapGene performed the expression of the vaccine-conjugated pET-28a(+) plasmid vector. The vaccine inserts are represented as a red circular portion within the plasmid vector backbone (black circle).

### Immune simulation

After a successful three-dose vaccine regime, there was a notable increase in the B-cell population for both V1 (Fig 9A) and V2 (Fig 9B), and the total amounts of B-cells remained active, indicating a sustained year-long immunity (Fig 9A and 9B). The T cell responses, including T_H_ and TC, were also evident for both V1 and V2 vaccines. The study also showed elevated expression of active T_H_ on day 60, which gradually decreased but sustained for nearly a year (S6 Fig). Furthermore, active T_C_ exhibited high-level expression after the post-vaccination regime and remained active for a year around (Fig 9C and 9D).

**Fig 9:** C-ImmSim predicted the immune simulations of the V1 and V2. The evolution of B-cell (A, B), cytotoxic T-cell (C, D), and Mφ (E, F) populations after three successive injections of the vaccine.

The innate immune response, including Mφ, NK, and DC-mediated immune responses, was also evident for V1 and V2. Both vaccines, V1 and V2, showed elevated levels of Mφ responses until 100 days of post-vaccination (Fig 9E and 9F), while NK showed one-year sustainable immune responses (S6 Fig). However, both vaccines showed reduced levels of DC activity (S6 Fig).

The article "Designing of an mRNA vaccine against high-risk human papillomavirus targeting the E6 and E7 oncoproteins exploiting immunoinformatics and dynamic simulation" was retracted in 2025. Reasons: compromised peer review; unreliable results or conclusions.

### mRNA structure prediction

The V1 mRNA exhibited an MFE score of -502.60 kcal/mol for optimum and -375.43 kcal/mol for centroid structure. Moreover, the V2 mRNA exhibited an MFE score of -450.90 kcal/mol for optimum and -329.52 kcal/mol for centroid structure. The thermodynamic free energy was predicted to be -534.60 kcal/mol and -475.73 kcal/mol, respectively. Further, the MFE structures of V1 and V2 were correlated with a frequency of 0.00% in each ensemble (Fig 10). Therefore, the mRNA structure of these designed vaccines will remain stable throughout the process of entry, transcription, and expression in the host [131, 132].

**Fig 10:** Predicted mRNA structures of the V1 and V2 by RNAfold web server. The MFE structures of the V1 and V2 are represented with the base pair probabilities (A, B) and the positional entropy (C, D), while the centroid structures of the vaccines are represented with the base pair probabilities (E, F) and the positional entropy (G, H).

## Discussion

Vaccination is a prerequisite for enhancing public health and boosting global well-being by protecting against HPV infection and its related health effects. There are six authorized HPV vaccines available, all of which are virus-like particles (VLPs) type vaccines, including three bivalent (Cervarix^®^, Cecolin^®^, and WalrinvaxV) [133–135], two quadrivalent (GARDASIL^®^ and Cervavac^®^) [136, 137], and one ninevalent (GARDASIL9^®^) vaccine [138–140]. The bivalent vaccines provide protection against HPV types 16 and 18, which have been associated with over 70% of cervical cancers [141–143]. Nevertheless, these vaccines cannot effectively cure pre-existing cancers since their mechanism of action involves the deployment of antibodies explicitly targeting the HPV capsid protein. This protein’s expression occurs before the virus’s release, making these vaccines less effective in preventing the formation of pre-existing lesions. Therapeutic vaccines, in contrast, elicit a cellular immune response instead of producing antibodies, which allows them to target and combat infected cells [144, 145].

Although VLPs imitate the molecular makeup of viruses, they do not possess the genetic material required for reproduction. As a result, they may not stimulate as strong of an immunological response as live attenuated or mRNA vaccines, especially in certain groups like the elderly or persons with weakened immune systems [41]. The advancements in vaccine research have shown that mRNA-based therapeutic agents, which are rapidly growing, may effectively tackle the challenges encountered in developing vaccines for infectious diseases and cancer [42, 43]. With its non-infectious and non-integrating nature, mRNA considered a superior vaccination choice compared to subunit, killed, live-attenuated, and DNA-based vaccines [44–47]. Also, the stability of mRNA in living cells can be influenced by various modifications and methods of delivery, as it is naturally broken down by cellular processes [44–47]. However, mRNA vaccines may be given by systemic delivery, which involves injecting the vaccine directly into the circulation, often through intravenous injections. Local injections, delivered directly at the target location, provide an alternative to systemic delivery and minimize adverse effects. Targeted delivery may be achieved by directly administering the medication into the specific tissue, such as by internodal injection. Hence, there is a diverse range of options for administering substances by intravenous, subcutaneous, intradermal, intramuscular, and intranodal routes [145, 146]. Multiple mRNA-based vaccines for cervical cancer are currently being experimented with in clinical and pre-clinical trials. In a recent study, an mRNA vaccine was developed targeting the E6 and E7 oncoproteins of HPV 16 and HPV 18. They found that the mRNA vaccine considerably triggered strong T-cell-mediated immune responses and substantially inhibited tumor development in both subcutaneous and orthotopic tumor-implanted mice models. Additionally, they discovered that the vaccine resulted in a large infiltration of immune cells into tumor tissues [147]. In another study, a notable mRNA-based vaccine was developed to target the HPV 16 late oncoproteins E6 and E7. In a preclinical model of HPV 16-associated lesion, the vaccine demonstrated a targeted adaptive immune response specific to the antigen [148]. Considering these, this study focuses on the reverse vaccinology technique to produce mRNA vaccines in response to the urgent public need for a vaccine against cervical cancer.

The article "Designing of an mRNA vaccine against high-risk human papillomavirus targeting the E6 and E7 oncoproteins exploiting immunoinformatics and dynamic simulation" was retracted in 2025. Reasons: compromised peer review; unreliable results or conclusions.

Here, we successfully developed two mRNA vaccines (V1 and V2) targeting the E6 and E7 oncoproteins of HPV 16 and HPV 18. The HTL, CTL, and B-cell epitopes were predicted and used in subsequent vaccine development using several bioinformatics tools. All the selected epitopes were further assessed for antigenicity, allergenicity, and toxicity. We then utilized several linkers and adjuvants to construct the mRNA vaccines with the selected epitopes. According to physicochemical properties, both the vaccines’ products were predicted as soluble proteins, which might be functionally stable under body conditions [127, 149]. The vaccines were also predicted to be basic in nature with the theoretical pI of 8.73 and 6.62 for the V1 and V2, respectively. The aliphatic index of the V1 and V2 were predicted to be 84.33 and 78.26, respectively, indicating the vaccines as hydrophobic proteins containing aliphatic side chains [127, 150]. The instability indices for vaccines V1 and V2 were expected to be 61.89 and 57.24, respectively, indicating their instability. The glitch was rectified during the assessment of their tertiary structures. It is crucial to consider the process of protein folding into its secondary and tertiary structures while developing an effective vaccine. Both the unfolded and folded proteins’ antigens are essential in protein-specific immune responses; hence, these are the prime targets for antibodies, which in turn mount in response to infections [151]. The predicted secondary and tertiary structures of the V1 and V2 were found satisfactory and reliable. The Ramachandran plot analysis also showed that most of the vaccines’ residues were within the preferred regions (94.5% for V1 and 87.1% for V2), conferring the structural integrity of the tertiary structures. Also, the Z score of the V1 and V2 indicated the stability of the vaccine structures with scores of -5.15 and -4.1, respectively, and ERRAT scores of the vaccines confirmed the quality of the V1 (92.771) and V2 (83.497) models.

To evaluate the possible association between the vaccines and TLRs on immune cells, a docking analysis was performed by Cluspro 2.0 utilizing human TLR-2 and TLR-4. According to this analysis, V1 exhibited a substantial affinity towards TLR-2 (lowest energy score of -1159.3 KJ/ml) and TLR-4 (lowest energy score of -1109.3 KJ/ml) receptors, where V2 exhibited a substantial affinity towards TLR-2 (lowest energy score of -1246.3 KJ/ml) and TLR-4 (lowest energy score of -1244.8 KJ/ml) receptors. According to the PBDsum, a total number of 25, 23, 17, and 38 hydrogen bonds were found within the “V1—TLR-2”, “V2—TLR-4”, “V2—TLR-2” and “V2—TLR-4” complexes, respectively.

Molecular dynamic simulation was also performed to validate the structural integrity of the vaccines and vaccine-TLR complexes. The analysis of RMSD values for V1 and V2 and their complexes with TLR-2 and TLR-4 indicated variable degrees of stability throughout the 100 ns simulation. While the RMSD values for V1 and V1—TLR-4 steadily increased over time, V1—TLR-2 exhibited a drastic initial increase, followed by a subsequent decrease in post-100 ns simulation time. The average RMSD values obtained at the end of the 100 ns simulation were 0.106 nm for V1, 0.116 nm for V1—TLR-2, and 0.081 nm for V1—TLR-4. The findings suggested that V1 adopted a more stable conformation when bound to TLR-4 than TLR-2. Conversely, the RMSD values for V2 and V2—TLR-2 showed steady growth, with V2—TLR-4’s fluctuation that eventually decreased after 100ns. The average RMSD for V2, V2—TLR-2, and V2—TLR-4 was 0.737 nm, 0.738 nm, and 0.860 nm, respectively. Therefore, the V2 was shown to be more stable when coupled with TLR-2 compared to TLR-4.

The article "Designing of an mRNA vaccine against high-risk human papillomavirus targeting the E6 and E7 oncoproteins exploiting immunoinformatics and dynamic simulation" was retracted in 2025. Reasons: compromised peer review; unreliable results or conclusions.

Furthermore, the RMSF analysis highlights distinct regional flexibility patterns, particularly evident in V1—TLR-2 compared to V1 and V1—TLR-4. With an average RMSF value of 0.80 nm, V1 was a bit flexible when it wasn’t tied to the TLRs. When V1 interacted with TLR-2, its flexibility was considerably reduced to 0.61 nm, which suggests that TLR-2 has a stabilizing impact on the V1 residues via its contact. With TLR-4, the RMSF value was lowered to 0.71 nm, reflecting a lesser degree of flexibility reduction than the TLR-2 interaction [152, 153]. On the other hand, V2—TLR-4 residues showed more altered RMSF values than V2 and V2—TLR-2. The motility pattern of V2 bound to TLR-4 exhibited more significant changes than its unbound state and its interaction with TLR-2, indicating enhanced flexibility and instability during the V2—TLR-4 interaction [154, 155]. Upon binding to TLR-2, V2 had reduced fluctuations, indicating a stabilizing influence of TLR-2 on V2 residues. The RMSF value decreased from 0.29 nm in the unbound state to 0.25 nm in the V2—TLR-2 complex, indicating that this interaction constrained the movement of V2, resulting in increased stability. In contrast, the interaction with TLR-4 significantly increased RMSF to 0.56 nm, indicating enhanced residue flexibility [152]. The increased flexibility in the V2—TLR-4 complex suggested a more unstable interaction, perhaps leading to functional consequences. The disparity in RMSF patterns between V2 associated with TLR-2 and TLR-4 indicated that TLR-2 more efficiently stabilizes the V2 domain, while TLR-4 binding leads to increased dynamic fluctuations and possible instability.

Additionally, the Rg values indicated higher structural compactness of V1 and V1—TLR-4 compared to V1—TLR-2, while V2—TLR-4 had a more fragile structure compared to V2 and V2—TLR-4. During the simulation, the Rg value of the V1—TLR-2 complex consistently surpassed that of both the unbound V1 and the V1—TLR-4 complex. The Rg for the unbound V1 was measured at 2.96 nm, but the Rg values for the V1—TLR-2 and V1—TLR-4 complexes were found to be 3.46 nm and 3.24 nm, respectively. The findings revealed that V1 has enhanced structural stability in the presence of TLR-4, suggesting a more efficient binding interaction. The Rg analysis for V2 concurrently revealed significant differences depending on its interaction with various TLRs. The unbound V2 had an Rg of 2.96 nm, indicating its very compact topology. Upon interaction with TLR-2, the Rg value increased to 3.79 nm, demonstrating a significant structural expansion that signifies a less compact shape relative to the unbound state. The V2—TLR-4 complex exhibited an Rg of 3.53 nm, indicating a more compact structure than V2—TLR-2 yet still more extended than the unbound V2. The significant enlargement seen in the V2—TLR-2 complex suggested that this receptor may elicit conformational alterations that disrupt the compact structure of V2 more than TLR-4 responses. In the post-100 ns simulation, the SASA values remained nearly identical for V1, V1—TLR-2, and V1—TLR-4, while V2 exhibited lower values compared to V2—TLR-2 and V2—TLR-4, indicating differences in surface accessibility. The V1—TLR-2 complex had the highest SASA value at 291.29 nm^2^, surpassing V1 (261.55 nm^2^) and V1—TLR-4 (275.51 nm^2^). The heightened solvent exposure in the V1—TLR-2 complex suggests enhanced flexibility or a conformational alteration. Although V1 exhibited minimal solvent exposure, the V1—TLR-4 complex had an intermediate SASA value, indicating a lesser extent of structural alteration. Conversely, V2 consistently showed lower SASA values than its complexes with TLR-2 and TLR-4. Initially, the SASA values for the V2—TLR-2 and V2—TLR-4 complexes were quite similar, suggesting comparable solvent exposure. However, by the end of the simulation, the V2—TLR-2 complex revealed the highest SASA value of 662.76 nm^2^, while the V2—TLR-4 complex recorded a substantial SASA of 643.99 nm^2^. In contrast, the unbound V2 had a SASA of 420.43 nm^2^. These results suggested that the binding of V2 to TLR-2 and TLR-4 leads to structural changes, increasing its exposure to the solvent.

The article "Designing of an mRNA vaccine against high-risk human papillomavirus targeting the E6 and E7 oncoproteins exploiting immunoinformatics and dynamic simulation" was retracted in 2025. Reasons: compromised peer review; unreliable results or conclusions.

The simulation run provided critical insights into the dynamic behavior of hydrogen bonds within the docked complexes, illustrating how molecular interactions evolve over time [48]. Initially, at 0 ns, the counts of hydrogen bonds were modest, with V1—TLR-2 at 10, V1—TLR-4 at 11, V2—TLR-2 at 13, and V2—TLR-4 at 16. As the simulation progressed to 25 ns, fluctuations in hydrogen bonding were observed. Notably, V2—TLR-4 exhibited a remarkable increase in hydrogen bonds, rising to 26, which may indicate enhanced stability or a stronger interaction with its ligand compared to the other complexes. The mid-simulation assessment at 50 ns highlighted continued variability, with V1—TLR-2 increasing its hydrogen bond count to 18 while V1—TLR-4 remained stable at 16. This stability in V1—TLR-4 might imply that the binding interactions are reaching an equilibrium state, while V1—TLR-2’s increase suggests ongoing adaptation in its binding environment. Conversely, V2—TLR-2’s reduction in hydrogen bonds to 12 indicates a potential weakening of its interaction, which may affect its overall stability and function. By the end of the simulation at 100 ns, the final counts revealed 21 hydrogen bonds for V1—TLR-2, 13 for V1—TLR-4, 15 for V2—TLR-2, and a striking increase to 36 for V2—TLR-4. The pronounced growth in hydrogen bonds for V2—TLR-4 suggests a strong affinity for its ligand, reinforcing the notion that this complex may represent a key target for further biochemical exploration [153, 156].

Codon optimization was employed to assess the expression of recombinant vaccines in the *E*. *coli* cloning vector, especially the K12 strain. The experimental results indicate that both vaccines showed substantial expression in the vector. The average GC content of the adapted V1 and V2 sequences were calculated as 51.88% and 51.63%, respectively, while both vaccines showed a CAI score of 1.0 each. After administering three doses of the vaccines, there was a significant increase in B-cell populations for both V1 and V2, indicating sustained immunity for a year. T-cell responses, including T_H_ and T_C_, were also observed for both vaccines, with elevated expression of active T_H_ cells on day 60 and sustained T_C_ activity post-vaccination. Additionally, innate immune responses, including Mφ, NK, and DC responses, were evident for both vaccines. Elevated Mφ responses were observed up to 100 days post-vaccination, while NK exhibited sustained immune reactions over a year. However, both vaccines showed reduced DC activity. The secondary structure predictions of the V1 mRNA vaccine revealed an optimal MFE score of -502.60 kcal/mol and a centroid structure score of -375.43 kcal/mol. Similarly, for V2, the MFE score was -450.90 kcal/mol for the optimal structure and -329.52 kcal/mol for the centroid structure. The thermodynamic free energy predictions were -534.60 kcal/mol and -475.73 kcal/mol for V1 and V2, respectively. Additionally, the MFE structures of both vaccines exhibited a correlation frequency of 0.00% within the ensemble, indicating a unique and stable structural conformation for each. Consequently, the mRNA structures of V1 and V2 are poised to maintain stability during entry, transcription, and expression in the host, ensuring their efficacy and functionality.

However, a notable limitation of this study is the inability to extend the simulation beyond 100ns because of lacking access to suitable machine. A longer trajectory, such as a 200ns simulation, would provide a more thorough investigation of ligand-receptor interactions, perhaps uncovering more stable or variable binding patterns over time. This constraint may have hindered the comprehensive observation of equilibrium states or prolonged binding behaviors. Finally, this work emphasizes the ability of the two mRNA vaccines against HPV 16 and HPV 18 to stimulate robust humoral and cellular immune responses against the virus. Considering the facts and potential findings of the study, further *in vitro* and *in vivo* analyses are strongly recommended. Therefore, our research will now focus on conducting further laboratory experiments to evaluate the efficacy and safety of the designed vaccines.

The article "Designing of an mRNA vaccine against high-risk human papillomavirus targeting the E6 and E7 oncoproteins exploiting immunoinformatics and dynamic simulation" was retracted in 2025. Reasons: compromised peer review; unreliable results or conclusions.

## Conclusion

We successfully designed two mRNA vaccines targeting the E6 and E7 oncoproteins of the high-risk HPVs: HPV 16 and HPV 18. Bioinformatics tools aided epitope selection, with subsequent structural assessments confirming stability and antigenicity. Docking analysis revealed strong interactions between vaccines and TLRs, crucial for immune activation. Molecular dynamics simulations highlighted the stability and flexibility of vaccine complexes. Codon optimization ensured efficient expression in *E*. *coli* vectors. After vaccination, sustained B-cell and T-cell responses were observed alongside innate immune activation. Secondary structure predictions confirmed stable mRNA structures, which are vital for vaccine efficacy. Overall, V1 and V2 vaccines exhibit promising characteristics for inducing robust and durable immune responses against HPV infections. Although this comprehensive evaluation provides crucial insights into the vaccines’ characteristics, *in vitro*, *in vivo*, and clinical trials are imperative to validate their efficacy, safety, and potential in combating HPV infection and preventing its associated cancer. This study will provide a solid foundation for further research, emphasizing the need for subsequent experimental validations and clinical investigations to ascertain the translational potential of these mRNA vaccines.

## Supporting information

S1 Fig The secondary structure of V1 and V2 predicted by SOPMA and GOR4. (TIF)

S2 Fig The secondary structures of V1 and V2 predicted by PSIPRED. The polarity of the vaccine is remarkable along with its hydrophobicity (A), whereas, the three-state structure prediction depicted the vaccine has enormous helical region (B).
(TIF)

S3 Fig Disulfide engineering of V1 and V2. The wild models of the V1 (A) and V2 (B) contain no disulfide bond, while the mutant V1 (C) and V2 (D) models contain two pairs (LYS 178- TYR 418, ALA 201-HIS 390, and GLY 244- ALA 344) and three pairs (GLY 46-ASP 98, GLY 89-ASP 136, and LEU 188- ALA 200) disulfide bond.
(TIF)

S4 Fig The generalized Born and surface area solvation (MM-GBSA) analysis of the V1 and V2. The illustration represents intermolecular interactions including van der Waals forces (VDW), electrostatic interactions (ELE), polar (GB), and non-polar (SA) components.
(TIF)

S5 Fig Hydrogen bond analysis. Interchain hydrogen bonds between TLR-2 and V1, TLR-4 and V1, TLR-2 and V2, and TLR-4 and V2 were depicted in red, yellow, green, and orange, respectively.
(TIF)

S6 Fig Immune simulation analysis of the V1 and V2 including helper T cell (TH) (A, B), natural killer cell (NK) (C, D), and dendritic cell (DC) (E, F) responses. (TIF)

S1 Table DiscoTope 2.0 predicted the discontinuous B-cell epitopes residues of the vaccine structure. (DOCX)
